The article "Network Blockchain Security Sharing Model Based on Fuzzy Logic" was retracted in 2023. Reasons: unreliable results or conclusions; concerns about the data; concerns about the peer review; concerns about the citations.

# Network Blockchain Security Sharing Model Based on Fuzzy Logic

**DOI:** 10.1155/2022/1509000

**Published:** 2022-04-30

**Authors:** Ming Li, Peng Xiao

**Affiliations:** ^1^School of Computer and Information Technology, Mudanjiang Normal University, Heilongjiang, China; ^2^First School of Clinical Medicine, Mudanjiang Medical University, Mudanjiang, Heilongjiang, China

## Abstract

In light of the continuous development of Internet technology, many problems involving network security based on the blockchain have also been observed gradually. In this paper, the existence forms of network security hazards based on the blockchain are explored to establish a network blockchain security sharing model based on fuzzy logic. In security sharing, network blockchains are often maintained by many parties. This poses new potential threats and challenges to privacy protection in these multiparty network blockchains. This paper proposes a research scheme for a network blockchain security sharing model based on fuzzy logic. The tampering of the protected network blockchain is prevented by blockchain, and the fuzzy logic algorithm is used to ensure its confidentiality. This solution allows the exchange in the protected network blockchain and the security of transaction information based on the fuzzy logic algorithm. According to the results of the experiments, this method can ensure security sharing of the network blockchain with high practicality and achieve the expected design effect.

## 1. Introduction

As Internet technology continues to develop, additions problems of network security have also emerged. Many network security incidents in different fields have occurred at home and abroad. The security issues that exist in the network blockchain can be broadly classified into three categories as the following: the security problems that occur during the operation of the Internet itself, the security problems that occur when the Internet is attacked from the outside, and the security problems that occur when the maintenance and management of the network are upgraded. With the threat of any type of security risk, the daily maintenance and management based on the Internet aim to keep the healthy, stable, and rapid development of the Internet [1, 2]. The security, confidentiality, integrity, and detection mechanism of the whole operating system or data application and the sharing process of the Internet face tremendous security risks due to the defects in the system security of users in the Internet operation process [3, 4]. Hence, it is crucial to design a blackchain-based network system for security sharing. A security sharing model consistent with current Internet and multimedia technologies is developed and designed to further improve the security system associated with the Internet and its data application process and ensure relevant data security. In this way, confidentiality and availability can be ensured for better usage. As an effective method for monitoring the security in the existing network, the network blockchain security sharing model (NBSSM) can greatly improve the control over the network operation security and the active defense capacity of the network.

The article "Network Blockchain Security Sharing Model Based on Fuzzy Logic" was retracted in 2023. Reasons: unreliable results or conclusions; concerns about the data; concerns about the peer review; concerns about the citations.

For the purpose of storing and protecting the network blockchain, it is highly attractive if the storage and protection applications for network blockchain can be migrated to the cloud, which will save resources and also have cost efficiency. However, this can also make it tricky to prevent network blockchain loss and privacy breaches and ensure information security. What's more, by storing network blockchains in the cloud, the complete control of people over their personal network blockchains is lost, which is required for the confidentiality, integrity, and privacy of the blackchain-based network [5, 6]. In addition to the challenges mentioned above, in some secure shared applications, it is often necessary for multiple actors to maintain the network blockchain (such as certificate authority) to protect the root keys of private certificates. How to address the information security problem in this case remains a top priority and also one of the most significant concerns in the field of security sharing. Ambiguous logic is the core technology applied in digital cryptocurrency systems (such as Bitcoin), and it is a type of technology that can establish a peer-to-peer trusted data network with centralized distributed storage. How to integrate ambiguous logic with the Internet of Things (IoT), information systems, and business forms to resolve the problem of security sharing of centralized data among networks, systems, and businesses to meet the demands of the energy Internet is an issue that has to be solved at present.

Hence, a network blockchain security sharing model based on the fuzzy logic algorithm is established in this paper. This model can be effectively used in the network blockchain security sharing model by using a centralized data naming method, which has solved the security problems that may arise in the use of Internet data information.

## 2. Algorithm and Methods

### 2.1. Fuzzy Logic Algorithm

Fuzzy logic allows the user to carry out the ciphertext-specific algebraic operation directly, obtain the result, and repeat the process on the results of plaintext encryption. According to security parameters, public and private keys are produced, where *pkskλpk* are used for encrypting the plaintext, and *sk* is used for for decrypting the ciphertext. It is assumed that the plaintext is *m* ∈ *Z*_*n*_, in which *n* stands for a relatively large positive integer; *Z*_*n*_ stands for the integer modulo *n* set. The encryption of *m* is expressed as *E*_*pk*_(*m*). In this way, the fuzzy logic has the following features:

(1) $$\begin{array}{c} E_{pk}\left(m_{1}+m_{2}\right)=E_{pk}\left(m_{1}\right)⊕E_{pk}\left(m_{2}\right),\\ E_{pk}\left(a\times m_{1}\right)=a⊗E_{pk}\left(m_{1}\right). \end{array}$$

In the above equation, *m*_1_ and *m*_2_ stand for the plaintexts to be encrypted, a stands for a constant.

The article "Network Blockchain Security Sharing Model Based on Fuzzy Logic" was retracted in 2023. Reasons: unreliable results or conclusions; concerns about the data; concerns about the peer review; concerns about the citations.

Based on the homomorphic features of the system, a number of practical and effective cryptographic algorithms can be constructed. In this paper, we focus on the security of multiparty networks. Due to its additive homomorphic feature and compliance with the threshold cryptosystem design, the threshold fuzzy logic algorithm is applied in the solution [7, 8].

This paper uses a fuzzy logic algorithm with the threshold of (*p*, *t*), where the private key *sk* is partitioned (*sk*_1_, *sk*_2_,…, *sk*_*p*_) and assigned to *p* parts so that each party holds an incomplete private key. Where a party wants to decrypt the ciphertext, it still needs the keys from at least (*t* − 1) parties.

Specifically, each party *i*(1 < *i* < *p*) needs to use its private key to calculate its partial decryption *c*_*i*_ in the decryption step, as shown in the following:

(2) $$\begin{array}{c} c_{i}=c^{2\Delta sk_{i}}. \end{array}$$

In the above equation, Δ=*p*!.

The fuzzy logic algorithm is an analytical method between maximum and minimum.

When *w*=(1,0,0, ⋯, 0), the following can be obtained:

(3) $$\begin{array}{c} F\left(a_{1},a_{2},\ldots ,a_{n}\right)=\max\left(a_{1},a_{2},\ldots ,a_{n}\right)=b_{1}. \end{array}$$

When active defense is analyzed, the fuzzy logic algorithm (“or” analysis) is shown as the following:

When *w*=(0,0,0, ⋯, 1), the following can be obtained:

(4) $$\begin{array}{c} F\left(a_{1},a_{2},\ldots ,a_{n}\right)=\max\left(a_{1},a_{2},\ldots ,a_{n}\right)=b_{n}. \end{array}$$

When active defense is analyzed, the fuzzy logic algorithm (“and” analysis) is shown as the following:

If *w*=(1/*n*, 1/*n*, 1/*n*,…, 1/*n*), the following can be obtained:

(5) $$\begin{array}{c} F\left(a_{1},a_{2},\ldots ,a_{n}\right)=\frac{1}{n}\sum_{i=1}^{n}a_{i}. \end{array}$$

The fuzzy logic algorithm equals to the arithmetic mean analysis.

The identification of variable weights in the fuzzy logic algorithm is closely related to the data information base. For the purpose of ensuring the data information security of the network based on the blockchain, a discretization method based on the Gaussian data distribution is adopted in this paper, and the data on the degree of freedom are subject to a weighting process, which can eliminate the security hazard.

The article "Network Blockchain Security Sharing Model Based on Fuzzy Logic" was retracted in 2023. Reasons: unreliable results or conclusions; concerns about the data; concerns about the peer review; concerns about the citations.

The set *μ* stands for the mathematical expectation of (1,2,…, *n*), and the weight vector assigned is *w*=(1/*n*, 1/*n*,…, 1/*n*); *σ* is the standard deviation of *μ* and weight vector w in (1, 2,…, *n*). Thus, the following can be obtained:

(6) $$\begin{array}{c} \mu_{n}=\frac{1}{n}\frac{n\left(n+1\right)}{2}=\frac{n+1}{2},\\ \sigma_{n}=\sqrt{\frac{1}{n}\sum_{i=1}^{n}{\left(i-\mu_{n}\right)}^{2}},\\ \omega^{\prime }=\frac{1}{\sqrt{2\pi \sigma_{n}}}e^{-{\left(i-\mu_{n}\right)}^{2}/2\sigma_{n}^{2}},\\ \omega =\frac{\omega^{\prime }}{\sum_{i=1}^{n}\omega^{\prime }}. \end{array}$$

When assessing *n* information systems, it is assumed that the evaluation set is *D*=(*d*_1_, *d*_2_,…, *d*_*n*_), in which *d*_*k*_(*k*=1,2,…, *m*) stands for the K-th evaluator, and the subjective judgments given in the form of evaluations are as the following: the utility value is *u*^(*k*)^=(*u*_1_^*k*^, *u*_2_^*k*^,…,*u*_*n*_^*k*^)^*T*^, the active defense analysis language assessment value is *S*=(*s*_0_, *s*_1_,…, *s*_*T*_), and the complementary judgment matrix for active defense analysis is *p*_(*k*)_=(*p*_*ij*_^(*k*)^)_*n*×*n*_. The information thus determined is turned into utility value [9].

### 2.2. Model Establishment

The blockchain-based network security sharing model is shown in Figure 1 as follows, from which it can be observed that in accordance with the constructed network blockchain security sharing model, it is responsible for the joint and private chain by virtue of the Internet system architecture [10, 11]. In this way, it can implement the transformation of the data information security management into the application of fuzzy logic algorithm to complete the storage of data information. In accordance with the distribution protocol in the interconnection network, it can achieve the peer-to-peer data information between the network security management and users, with the details described in the following sections.

#### 2.2.1. Uniform Naming Method and Centralized Management of the Internet Data Information

According to the proposed system, the enterprise-related data and unified resource standards can be used to build the network of shared data information in a secure manner based on the blockchain, and scalable application systems can be achieved through the application of the technology [12, 13]. The indexing of local naming and data information can be quickly implemented in the Internet environment, which has provided a method for information data naming and indexing of the relevant security data information that can be extended. In this way, users can have access to the relevant open data, laying a sound foundation for sharing reliable Internet data information.

The article "Network Blockchain Security Sharing Model Based on Fuzzy Logic" was retracted in 2023. Reasons: unreliable results or conclusions; concerns about the data; concerns about the peer review; concerns about the citations.

#### 2.2.2. Storage of the Internet Secure Distributed Data

Blockchain is used as the foundation for the network blockchain for the storage of valid data, and the access authority is restricted by using authorized encryption. In addition, according to the actual business demands and features, the storage of distributed data is completed at the edge of the Internet, and the issue of data cache management is also a problem of sharing the secure data in the network.

#### 2.2.3. Efficient Data Distribution Protocols That Can Implement Autonomy and Equality

The essence of the network security data sharing based on the fuzzy logic algorithm is that it can implement the peer-to-peer sharing network P2PICN based on the Internet data. With regard to the network blockchain security studied in this paper, it is mainly used to implement the naming and analysis of the blockchain data in the process of information data delivery, in which centralized DNS domain name resolution services are required for the purpose of allowing effective reliable transmission of the network blockchain data.

The security sharing and risks based on the real-time security monitoring platform of the network blockchain is put forward. The structure of the network blockchain security sharing system is shown in Figure 2. The monitoring system is divided into four modules: rule input, traffic acquisition, data analysis, and database [14].

In the network security sharing system based on the blockchain, the business acquisition system filters and aggregates the network business through thousands of real-time network business as per the rules of the input system, saves the valid data in the database, and provides them to the data analysis system for further processing. Valid data are processed in the analysis system, and the changes in the network business and the adjustment of distribution information are shared accordingly. The network blockchain securely shares the actions of the network.  Figure 3 illustrates the process flow of the system network security sharing system based on the blockchain [15].

IP packets are analyzed and consolidated to obtain source, destination IP, data volume, application protocol, and other information required. The advantage of doing so is that it does not change the network structure, increase the network load, or take up any network resources [16]. In other words, it is independent of the waiting time of the network and thus has no impact on the network usage by the users.

The article "Network Blockchain Security Sharing Model Based on Fuzzy Logic" was retracted in 2023. Reasons: unreliable results or conclusions; concerns about the data; concerns about the peer review; concerns about the citations.

In this paper, the fuzzy logic is used to implement Sniffer based on a relatively simple method, in which only the grouping above the IP layer is cut, thus the frame information is not included. In this way, several special requirements can be met [17]. The analysis of the current network business network blockchain security sharing system suggests that in the whole network business, any change in the monitoring platform business of the immersive virtual reality (VR) network in real time is essential that of the network business as a whole, which can reflect the real-time monitoring platform business of the workstation and thus can be used to analyze the network performance instead of the general business. In other words, the service information can be obtained based on the raw socket [18]. It can be seen from Figure 4 that the cluster head vector set of multi-internet network sensing data nodes is established by initializing the network with a link monitoring system of monitoring nodes based on a multi-internet network. The dataset is divided into multiple 2D subregions Ak by time window width, where Ak stands for a 2D information entropy set that complies with A1 cell and A2 cell, cell Ak = *A*. *D*_*n*_|*d*_*n*−max_ − *d*_*n*−min_| · (1/*K*) and the channel assignment layout for two nodes of relay based on the Internet network security device is as shown in Figure 4.

### 2.3. Experiments and Result Analysis

This paper uses the fuzzy logic algorithm to predict network security, which has improved prediction accuracy. The experiment is conducted with the data from network security and dynamic weekly reports as the experimental data: the number of hosts infected with viruses, websites being tampered with, backdoor websites being implanted, forged web pages on domestic websites, and new information security vulnerabilities as evaluation indicators. In this way, the modern network security situation can be reflected in a comprehensive manner, which can be used as a basic index for assessing the weekly network security situation. The cybersecurity data from issue 1, 2015, to issue 7, 20l7, are used to carry out this experiment.

As shown in Figure 5, the NBSSM hypervisor library is responsible for creating, adding, deleting, configuring, and protecting the data of NBSSM. In the data acquisition process, NBSSM formats the detection data in accordance with a uniformly configured data format. In the data processing, NBSSM carries out the data processing such as merging, cross-referencing, and filtering on the normalized data according to the rules and saves the results in the network repository.

The article "Network Blockchain Security Sharing Model Based on Fuzzy Logic" was retracted in 2023. Reasons: unreliable results or conclusions; concerns about the data; concerns about the peer review; concerns about the citations.

After the design and development of the network blockchain security sharing model, as the security sharing model design in the specification is activated, it is necessary to run further tests on the performance of the system. Thus, other operations can be developed normally. The occupancy of system CPU and memory is used as an evaluation indicator. After the system is running, its CPU and memory occupancy is tested. The results show that its CPU occupancy is below 20%, and the memory occupancy is below 120 M in the implementation environment. This suggests that the designed security sharing model has little interference in the normal performance of the other Internet services.  Figure 6 indicates the test results of the performance metrics of the Internet after 10 h of execution based on the activated network blockchain security sharing model. In general, it has a mean Internet CPU usage rate of less than 3%, a peak usage of below 12%, a virtual memory of 100 MB, and a used Internet memory (workgroup) of 108 MB. After the security sharing model is activated, the normal business operation of the computer is not affected in any way, shape, and form. Since December 2018, the security sharing model has been applied in multiple cases after configuration and commissioning. In accordance with the results of the trial run for 6 months, the network blockchain security sharing model can protect Internet security perfectly. In addition, it is easy and practical to operate the system, which can achieve the expected effect and facilitate the further rollout of the application.

## 3. Discussion

With the continuous development of Internet network, due to the outbreak of various incidents of information data leakage, users of the Internet network have higher and higher demands for the security of personal information. The establishment of a secure environment for the information on the Internet network can protect the security of diverse data effectively. To this end, efforts in the construction of information security based on the traditional information security protection measures should be enhanced continuously. The most effective way to protect cybersecurity is to proactively enhance security sharing of network information for users. Internet network firewall is a highly effective protection technology. Various security levels are set so that illegitimate users in the external network environment can hardly invade the network system, which has played a very significant role in fully ensuring the security of information within the Internet network. In the cybersecurity threat information sharing model, the decentralization and anonymity features of blockchain technology are used to protect the privacy information of organizations involved in the cybersecurity threat information sharing and the related organizations. In addition, it is conducive to facilitate the reasoning and analyze the complete cyber-attack chain. Based on the traceability of blockchain, it is possible to trace back to the threat source in the attack chain, and the smart contract mechanism can be used to implement automatic alert response to any cyber threats.

The article "Network Blockchain Security Sharing Model Based on Fuzzy Logic" was retracted in 2023. Reasons: unreliable results or conclusions; concerns about the data; concerns about the peer review; concerns about the citations.

## 4. Conclusion

For the purpose of addressing hacker attacks, natural disasters, Internet viruses, and other security issues, this paper designed a protection system for cybersecurity based on the blockchain. The system has three layers as follows: application, core, and hardware. After the security sharing model designed in this paper is applied, 20% of CPU utility can be saved in normal operation conditions, and the memory consumption can be kept at less than 120 M without affecting the stable operation of the Internet.

## Figures and Tables

**Figure 1:** Security sharing model for network blockchain based on the fuzzy logic.

**Figure 2:** Architecture of the network blockchain security sharing system.

**Figure 3:** System flow.

**Figure 4:** Layout of the assignment of the double-layer relay node channel for Internet network security.

**Figure 5:** Data acquisition and processing based on NBSSM.

**Figure 6:** Test results of blockchain security sharing model performance based on the blockchain.

## Data Availability

The data used to support the findings of this study are available from the corresponding author upon request.
